# Stressors of Nursing Interns and Their Influencing Factors: A Cross-Sectional Study

This article has been retracted.

**DOI:** 10.1155/2021/3561628

**Published:** 2021-10-14

**Authors:** Xiaoqing Wang, Yu Han, Runyu Chai, Rong Chai

**Affiliations:** Qilu Hospital, Cheeloo College of Medicine, Shandong University, Jinan 250012, Shandong, China

## Abstract

**Objective:**

It is still unknown whether the stress level and stressors in Chinese nursing interns are influenced by teacher-related factors. This research was carried out for better understanding of the stress in nursing interns and distribution of stressors during their clinical practice and targeted measures to unwind the stress of nursing interns.

**Methods:**

A questionnaire survey, titled *Questionnaire on Stressors of Nursing Interns during Clinical Practice*, was conducted on nursing interns at a 3A Grade Hospital in Shandong Province. Characteristics of the nursing interns and stressors of nursing interns were collected. A multiple-linear regression model was used to explore the influencing factors of nursing interns' scores.

**Results:**

A total of 132 nursing interns were investigated in this study, and the overall stress scores were calculated. The stressors during the internship include the nature and content of the job, role orientation, workload, conflict between study and work, practice preparation, and interpersonal relationships. Gender, education level, instructor encouragement, and parents engaged in the medical industry were adjusted in the multiple-linear regression model as covariates. All of these factors had significant impacts on the scores of stressors (*P* < 0.05), with the partial regression coefficient values of 13.38, −10.52, −5.02, 3.4, −9.89, −14.77, and −15.83 for factors like female, undergraduates, graduate students, never obtained encouragement from teachers, obtained encouragement from teachers occasionally, obtained encouragement from teachers frequently, and parents engaged in the medical industry, respectively.

**Conclusion:**

The stressors of nursing interns are mostly work-wise, and teachers' encouragement is an important protective factor for nursing interns to reduce stress. Therefore, clinical instructors should take targeted measures in teaching methods and work arrangements according to the needs of interns.

## 1. Introduction

Clinical nursing practice is an important link of nursing interns' transition from theoretical learning to nursing practice, where nursing interns begin to face various patients and perform actual clinical nursing operations in an unfamiliar environment and can feel stressed about it. Excessive pressure may bring multiple negative effects to nursing students, such as reducing their confidence and learning enthusiasm, and affect their intention to engage in nursing occupation [1–3]. Nursing interns, mostly between 20 and 25 years of age, have strong learning ability and potential, but their ability to cope with stress and the ability to digest the negative effects of stress still need to be improved [4, 5]. Therefore, it is necessary to investigate the stressors in the clinical practice of interns, correctly recognize the psychological activities of interns, and take effective countermeasures to help nursing students maximize the positive effects of stress and reduce the negative effects of stress. In this way, nursing trainees are able to transform pressure into motivation, adapt and integrate into the work environment, and develop excellent professional skills. This is also the fundamental guarantee for the smooth development of nursing work [6, 7].

Previous research has explored the main root cause of stress and target strategies [8]. However, the results are controversial. The stress may come from work, life, or other aspects [8]. Moreover, there are very few studies on Chinese nursing interns, and whether the level of stress is influenced by teacher-related factors is still unknown. Based on these reasons, we hypothesized that the stress in Chinese nursing interns is mainly work-wise and explored the influencing factors of stress.

Using data from a 3A Grade Hospital in Shandong Province, in this study, we aim to identify the overall stress and the distribution of stressors during the clinical nursing practice, explore the influencing factors of the stress, and provide a basis for taking targeted measures to reduce the stress of nursing interns.

## 2. Methods

### 2.1. Study Design and Participants

A questionnaire survey was conducted for nursing interns in a 3A Grade Hospital in Shandong Province through questionnaire design, distribution, collection, and summary. Through data analysis, the overall stress and the distribution of stressors during the clinical nursing practice were explored, which provides a basis for taking targeted measures to reduce the stress of nursing interns.

The nursing interns who joined the 3A Grade Hospital of Shandong University in 2019 and volunteered to participate in this survey were selected for the questionnaire survey. During the survey, 160 questionnaires were issued, 150 questionnaires were returned, 18 questionnaires that were filled in irregularly or unclearly were rejected, and 132 valid questionnaires were collected, with the recovery rate of 93% and the effective rate of 88%. This study was approved by the Ethical Committee of the Qilu Hospital of Shandong University (Jinan, China).

### 2.2. Measurement

1. Characteristics of the nursing interns: on the basis of reference to the relevant literature, we have designed and formulated a survey on the general situation of interns, including age, gender, family income, whether serve as a class leader, education background, etc.
2. Questionnaire on stressors of nursing interns: this research as made with reference to the questionnaire of the stressors of nursing interns developed by Zhang et al. [9] and is based on the actual situation of Shandong University Qilu Hospital and other measurement tools for the stress of nursing interns [10, 11]. It was suitable for the stress evaluation of nursing interns. The content of the questionnaire includes 6 dimensions and 40 entries: nature and content of the job (9 entries), workload (5 entries), practice preparation (5 entries), interpersonal relationships (8 entries), conflict between study and work (9 entries), and role orientation (4 entries). The 5-point Likert scale was utilized for the assessment, with 1 point to 5 points for no pressure, mild pressure, moderate pressure, heavy pressure, and extremely heavy pressure, respectively. The higher the score, the greater the stress. The scale tested the retest reliability and factor structure, with good reliability and validity. The Cronbach *α* was 0.81, the correlation between the scores of overall stress and the scores of stress in various dimensions was between 0.56 and 0.73, and the retest reliability was 0.79. The factor loading ranged from 0.663 to 0.955, with a comparative fit index (CFI) equal to 0.821 and a root mean square residual (RMR) equal to 0.078, respectively. Supplementary Table S1 presents the detailed results.

### 2.3. Investigation Method

With the assistance of the head nurse of each department, we contacted the heads of the nursing interns before the questionnaire survey and obtained the informed consent of the nursing interns. The questionnaire was distributed to groups of nursing interns, and the precautions were explained to them. We checked the completed questionnaires and kept valid questionnaires after screening out invalid questionnaires.

### 2.4. Statistical Method

Statistical description and analysis were performed by using SPSS 22.0. The statistical description of data was conducted. The count data were expressed in frequency and percentage, and the measurement data were expressed in mean and standard error. The overall pressure score comparison between the two samples was implemented via the *t*-test. The analysis of the scores of overall stress and stress in various dimensions was conducted by multiple-linear regression analysis, with the inspection level of *α* = 0.05.

## 3. Results

### 3.1. General Demographic Characteristics of the Nursing Interns

In this survey, the age of interns was mostly between 20 and 25, accounting for 78.79% of all. The proportion of female nursing staff reached 81.06%, and that of nursing staff with a bachelor's degree or above was 59.09%. There were 32.58% of interns who were the only child of their families, and 63.64% of interns came from rural areas. The single-factor statistical test found that gender, education, instructor's encouragement, and parents engaged in the medical industry were related to the score of overall stress (*P* < 0.05). Other general demographic characteristics are shown in Table 1.

### 3.2. Scores of Stressors of the Nursing Interns

Dimensions of overall stress (109.89), nature and content of the job (27.98), workload (13.89), practice preparation (13.21), interpersonal relationships (20.20), conflict between study and work (23.33), and role orientation (11.26) were scored (see Table 2 for more details).

Table 3 shows the scores of top ten stressors. The entries with high scores are as follows: the patient's condition changes dramatically or dies when the doctor or the instructor is not present; needlestick injuries at work; nursing patients with AIDS, tuberculosis, hepatitis B, hepatitis C, etc.; patient death; nursing patients with violent tendencies; an overwhelming amount of work and physical exhaustion; irregular working hours and working in middle and night shifts and holidays; worries about not finding a satisfactory job; doing nonnursing jobs which are mostly trivial things; seeing patients suffering from illness. It can be seen that the stressors were mostly related with the nature and content of the job, as six of the top ten entries belonged to the dimension of nature and content of the job; the next included the workload, conflict between study and work, and role orientation.

### 3.3. Multiple-Linear Regression Analysis of the Scores of Overall Stress and Stress in Various Dimensions

A multiple-linear regression analysis of the scores of overall stress and stress in various dimensions was conducted. The results showed that gender, education, instructor encouragement, and parents engaged in the medical industry had a significant impact on the score of overall stress (*P* < 0.05) (see Table 4 for details).

## 4. Discussion

In this cross-sectional study, using a questionnaire survey, we evaluated the levels of overall stress in Chinese nursing interns, identified the distribution of stressors, and used multiple-linear regression to explore the influencing factor of the stressors. The main stress was work-wise, while the top three stressors were “the patient's condition changes dramatically or dies when the doctor or the instructor is not present,” “needlestick injuries at work,” and “nursing patients with AIDS, tuberculosis, hepatitis B, hepatitis C, etc.”. And, we found gender, educational level, encouragement from teachers, and the occupation of parents were all important influencing factors of stress, emphasizing that more attention should be paid to nursing interns and more encouragement from teachers should be provided which may reduce the nursing interns' stress.

Seley, the father of stress science, believes that stress is a human nonspecific response caused by stimulation in the environment, which unselectively affects all systems or most systems of the body [12]. Nursing interns are students who have just left campus for work and often bear great psychological stress from work and complex interpersonal relations that are different from the academic study in colleges [13, 14]. Zheng et al. [15] showed that the stress in most nursing interns is at a medium level. Sun et al. [16] found that nursing interns were under high work pressure during their first internship. When nursing interns work for the first time, the complexity of nursing environment will cause stress for them and various factors will bring difficulties in clinical practice, which affect the quality of clinical practice and nursing, thus affecting the confidence of nursing interns in nursing specialities [17–20]. Our study demonstrated that the nursing interns generally had a medium or high level of stress, which is in line with previous research studies [17–20].

Liang et al. [21] found that the stress of nursing interns who are starting out mainly includes the fear of mistakes and the uncertainty about decisions on nursing practice decisions; overload and shift work; huge burden and unfamiliar work culture; self-evaluation on whether to take up the nursing occupation; solutions to problems; control of emotions; and exploration for a right way for themselves. In this study, the stressors with scores from high to low were as follows: nature and content of the job, role orientation, workload, practice preparation, interpersonal relationships, and conflict between study and work. The stressors were mostly related to the nature and content of the job, as six of the top ten entries belonged to the dimension of nature and content of the job; the next included the workload, conflict between study and work, and role orientation. This result is similar to other findings. Shaban et al. [22] studied 181 nursing interns at two Jordanian universities, which showed that their stressors are mainly from the operational and clinical environment. Chan et al. [23] explored the stress of nursing undergraduates in Hong Kong and their coping strategies, which suggested that their stress is at a moderate level and the most common stressors were the lack of professional knowledge and skills.

The multiple-linear regression analysis of the scores of overall stress and stress in various dimensions showed that gender, education, instructor's encouragement, and parents engaged in the medical industry had significant impacts on the scores of stressors. The stressor score of male nursing interns was significantly lower than that of female nursing interns, and the stressor score of undergraduate nursing interns was lower than that of junior college students, which was consistent with the results of other studies [16, 24]; that is, the higher the education level, the less the work pressure. At present, there is little research on the correlation between the teaching behavior of clinical instructors and the stress in nursing interns. However, in this study, the number of clinical instructors encouraging nursing interns significantly reduced the stressors of nursing interns, which suggests that clinical instructors can further enrich the communication and teaching methods to reduce the stress of nursing interns. Although the differences in overall stressor scores across birthplaces were not statistically significant, studies have shown that [24] the psychological stress faced by urban students and rural students is significantly different. Urban students face more emotional and spiritual pressure, while rural students are mainly worried about employment, living consumption, and other practical problems. Hence, in the practice process, clinical instructors should take different care and stress release methods for different types of psychological stress [25].

There are some important strengths in this study. Using a questionnaire survey, we assessed the overall stress in Chinese nursing interns and identified the important stressors. This may be a basis of strategies to reduce the nursing interns in China. We also explored the influencing factors of stress to make target strategies. On the other hand, there are some limitations we should acknowledge. Firstly, this cross-sectional study does not consider the change pattern of stress; further study should explore the trends of stress in Chinese nursing interns. Secondly, the covariates we used in multiple-linear regression may be insufficient. Further potential influencing factors should be explored. Finally, the current study was a cross-sectional study based on Chinese nursing interns in Shandong Province, suggesting our study may not be generalizable to other populations.

## 5. Conclusion

To sum up, the stressors of nursing interns were mostly related to the nature and content of the job, and teachers' encouragement is an important protective factor for nursing interns to reduce stress. Thus, clinical instructors should take targeted measures in teaching methods and work schedules according to the needs of nursing interns to maintain the stress of nursing interns at a reasonable level.

## Figures and Tables

**Table 1:** General demographic characteristics of the nursing interns.

Demographic characteristics	Group	Number of people (%)	Stressor score	*P*
Age (years)	20∼25	104 (78.79)	110.94 (30.87)	0.379
	25∼30	28 (21.21)	105.96 (27.56)	

Gender	Male	25 (18.94)	98.48 (25.46)	0.035
	Female	107 (81.06)	112.55 (30.66)	

Education	Associate's degree	54 (40.91)	108.07 (29.95)	0.036
	Bachelor's degree	74 (56.06)	112.03 (30.81)	
	Master's degree	4 (3.03)	94.75 (17.46)	

Only child	Yes	43 (32.58)	105.42 (33.34)	0.223
	No	89 (67.42)	112.04 (28.45)	

Class cadre	Yes	43 (32.58)	104.67 (29.11)	0.257
	No	89 (67.42)	112.40 (30.50)	

Clinical practice time	≤3	3 (2.27)	97.00 (20.66)	0.740
	3∼6	25 (18.94)	114.76 (28.90)	
	6∼12	98 (74.24)	108.92 (30.08)	
	>12	6 (4.55)	111.83 (43.16)	

Birthplace	City	48 (36.36)	106.94 (33.67)	0.418
	Countryside	84 (63.64)	111.57 (28.03)	

Introversion	Yes	59 (44.70)	111.57 (28.03)	0.831
	No	73 (55.30)	109.21 (30.42)	

Family income (yuan/month)	≤1000	14 (10.61)	101.93 (36.20)	0.480
	1000∼2000	47 (35.61)	111.81 (25.48)	
	>2000	71 (53.79)	110.18 (31.90)	

Parents engaged in the medical industry	Yes	19 (14.39)	96.74 (27.77)	0.041
	No	113 (85.61)	112.10 (30.10)	

College preference	Voluntary choice	67 (50.76)	106.94 (27.09)	0.542
	Others' influence	59 (44.70)	113.31 (32.85)	
	Alternative major choice	6 (4.55)	109.17 (37.18)	

Instructor's encouragement (time/week)	Never (0)	45 (34.09)	114.29 (30.08)	0.048
	Occasionally (1∼2)	56 (42.42)	103.94 (21.73)	
	Regularly (≥3)	31 (23.48)	97.64 (40.90)	

**Table 2:** Scores of stressors of the nursing interns (mean ± SD).

Dimension	Entry	Total score of all dimensions	Average score of all dimensions
Nature and content of the job	9	27.98 ± 7.21	3.11 ± 0.80
Workload	5	13.89 ± 4.32	2.78 ± 0.86
Practice preparation	5	13.21 ± 4.36	2.64 ± 0.87
Interpersonal relationships	8	20.20 ± 7.05	2.53 ± 0.88
Conflict between study and work	9	23.33 ± 8.03	2.59 ± 0.89
Role orientation	4	11.26 ± 4.30	2.81 ± 1.07
Total	40	109.89 ± 30.16	2.75 ± 0.75

**Table 3:** Scores of top ten stressors (mean ± SD).

Stressors	Dimensions	Scores
The patient's condition changes dramatically or dies when the doctor or the instructor is not present	Nature and content of the job	3.63 ± 1.11
Needlestick injuries at work	Nature and content of the job	3.58 ± 1.06
Nursing patients with AIDS, tuberculosis, hepatitis B, hepatitis C, etc.	Nature and content of the job	3.56 ± 1.06
Patient death	Nature and content of the job	3.28 ± 1.17
Nursing patients with violent tendencies	Nature and content of the job	3.24 ± 1.11
An overwhelming amount of work and physical exhaustion	Workload	3.05 ± 1.12
Irregular working hours and working in middle and night shifts and holidays	Workload	3.00 ± 1.16

Worries about not finding a satisfactory job	Conflict between study and work	2.95 ± 1.15
	Role orientation	

Doing nonnursing jobs which are mostly trivial things	Role orientation	2.92 ± 1.14
Seeing patients suffering from illness	Nature and content of the job	2.85 ± 0.97

**Table 4:** Multiple-linear regression analysis of the score of overall stressors.

		Regression coefficient	Standard error	*t*	*P*
Constant term		111.12	7.57	14.68	<0.001

Gender	Male	—	—	—	—
	Female	13.38	6.54	2.05	0.043

Education	Associate's degree	—	—	—	—
	Bachelor's degree	−10.52	5.34	−1.97	0.047
	Master's degree	−5.02	16.18	−0.31	0.757

Instructor encouragement	Never	3.43	1.64	2.09	0.038
	Occasional	−9.89	5.94	−1.67	0.099
	Regularly	−14.77	6.70	−2.21	0.029

Parents engaged in the medical industry		−15.83	7.78	−2.03	0.044

## Data Availability

The data used to support the findings of this study are available from the corresponding author upon request.

## Supplementary Materials

Supplementary Materials Supplementary Table S1 presents the results of factor structure. Obviously, the factor loading ranges from 0.663 to 0.955.
